# The protective effects of Olmesartan against interleukin-29 (IL-29)-induced type 2 collagen degradation in human chondrocytes

**DOI:** 10.1080/21655979.2021.1997090

**Published:** 2022-01-11

**Authors:** Yunlong Liu, Junyi Liu, Yan Ma, Yongyong Zhang, Qiong Chen, Xin Yang, Yanchun Shang

**Affiliations:** a Department of Knee Surgery, Luoyang Orthopedic-Traumatological Hospital of Henan Province, Zhengzhou, China; b Lab of Molecular Biology, Luoyang Orthopedic-Traumatological Hospital of Henan Province, Zhengzhou, China; c Department of Medicine, Affiliated Cancer Hospital of Zhengzhou University, Henan Cancer Hospital, Zhengzhou, Henan, China

**Keywords:** Osteoarthritis, IL-29, Olmesartan, extracellular matrix

## Abstract

Osteoarthritis (OA) is a cartilage degenerative disease commonly observed in the elderly population and is pathologically characterized by the degradation of the cartilage extracellular matrix (ECM). Matrix metalloproteinases (MMPs) and a disintegrin and metalloproteinase with thrombospondin motifs (ADAMTSs) are critical enzymes involved in the degradation of ECM. Olmesartan is an inhibitor of the angiotensin II receptor developed for the treatment of hypertension, and recent studies show that it exerts anti-inflammatory effects in arthritis. The present study aimed to investigate the mechanism of the protective effect of Olmesartan on cartilage ECM degradation. Interleukin-29 (IL-29) is a novel inflammatory mediator involved in the inflammation and degradation of cartilage in OA, and human T/C-28a2 cells treated with it were the inflammatory model *in vitro*. We found that the degradation of type 2 collagens and aggrecans was induced by IL-29, accompanied by the upregulation of MMPs and ADAMTSs, but the presence of Olmesartan significantly ameliorated these increases. In addition, Olmesartan abolished IL-29- induced oxidative stress and elevated the expression level of TNF receptor-associated factor 6 (TRAF-6). Mechanistically, we showed that Olmesartan suppressed IL-29- caused inhibitor kappa B α (IκBα) expression and nuclear translocation of nuclear factor kappa-B (NF-κB) p65, indicating it suppressed the activation of the NF-κB pathway. Collectively, our data reveal that Olmesartan exerted a protective function on IL-29- induced type 2 collagen degradation in human chondrocytes.

## Introduction

Osteoarthritis (OA) is a common clinical joint disease, and its risk factors include age, gender, weight, and trauma. Therefore, OA is regarded as a chronic and systemic degenerative disease [1]. In China, the overall morbidity of OA is approximately 15% and the prevalence elevates significantly with age [2]. The clinical characteristics of OA include slowly progressing joint pain, stiffness, swelling, limited flexion and extension, and joint deformity. At their advanced stages, these syndromes significantly impact the daily lives of the afflicted [3]. Currently, the pathological mechanism underlying OA remains unclear. The main pathological changes of OA are the loss of articular cartilage and subchondral sclerosis. Under pathological conditions, the balance between the degradation and synthesis of extracellular matrix (ECM) in chondrocytes is disrupted in OA cartilage tissues, contributing to the apoptosis of chondrocytes and loss of articular cartilage. The main components of the cartilage matrix are type II collagens and aggrecans. A reticular structure is formed by type II collagens while the aggrecans intersperse in the reticular structure. The unique three-screw structure of type II collagens provides the skeleton and elasticity for the articular cartilage and aggrecans to exert lubrication and compression functions by accumulating large amounts of water and metal ions [4]. The etiology of OA includes multiple factors, cytokines, gene regulation, molecular signaling, free radical theory, and metalloprotease theory [5]. Recently, the role of metalloprotease has been extensively investigated by OA scientists. The degradation and metabolism of ECM in chondrocytes are the leading cause of OA, and are closely associated with the malfunction of collagenases and aggrecanases. Matrix metalloproteinases (MMPs) are regarded as the classic enzymes involved in the degradation of collagens and aggrecans. In recent years, the A disintegrin and metalloproteinase with thrombospondin motifs (ADAMTS) family has been reported to play a critical role in the pathogenesis of OA. Among the collagenases and aggrecanases involved in the degradation of ECM during OA, MMP-1, MMP-13, ADAMTS-4, and ADAMTS-5 play major roles [6]. Therefore, the agents targeting collagenases and aggrecanases have been considered an effective approach to treat OA.

NF-κB is the master transcription factor involved in inflammatory processes and plays a critical role in OA chondrocytes and related signaling pathways [7]. Interleukin family cytokine-mediated signal transduction starts with the cytokine binding to its receptor and forming the receptor/MYD88-IRAK module. When IRAK kinases are phosphorylated, the complex recruits tumor necrosis factor–associated factors (TRAFs). TRAFs are a family of proteins that transduce signals from various immune receptors. TRAF6 is a pivotal factor of the TRAFs family of proteins. It binds to a receptor complex and mediates the activation of the IκB kinase (IKK) complex [8]. Activated IKK phosphorylates IκBα and promotes its degradation, thus releasing NF-κB p50 and NF-κB p65 subunits. Their nuclear translocation thereafter is the central step in the activation of NF-κB [9].

Olmesartan was originally developed by Daiichi-Sanyo and approved by the U.S Food and Drug Administration (FDA) in April of 2002 for the treatment of hypertension. In August 2006, Olmesartan was approved for marketing in China under the trade name Olrnetec [10,11]. Olmesartan exerts vasoconstriction and reduction of aldosterone secretion by specifically blocking angiotensin II and binding to the angiotensin 1 receptor located on vascular smooth muscles to suppress the production of renin [12]. Recently, the anti-inflammatory effects of Olmesartan have been reported [13,14]. Interleukin-29 (IL-29) is a newly identified inflammatory mediator belonging to a large IL-10 family. IL‐29 has emerged as a critical inflammation mediator in inflammatory autoimmune diseases [15]. A recent study shows that IL-29 plays a role in rheumatoid arthritis (RA) and is also involved in the pathogenesis of OA. Indeed, IL-29 protein levels are much higher in OA patients than those in healthy subjects. IL-29-induction stimulates inflammation and cartilage degradation by activating nuclear factor-κB (NF-κB) in OA synovial fibroblasts (FLS) [16]. Thus, IL-29 is considered a novel mediator of the inflammation and degradation of cartilage in OA. The treatment choice for OA remains very limited, and it is in our interest to explore if Olmesartan exhibits anti-inflammatory effects in activated chondrocytes. The present study is designed to investigate the potential protective effects of Olmesartan on OA using the IL-29-treated chondrocytes.

## Materials and methods

### Cell culture and treatments

Human T/C-28a2 chondrocytes were obtained from ATCC (Rockefeller, USA) and cultured in Dulbecco’s Modified Eagle Medium (DMEM) (Hyclone, Logan, USA) supplemented with 10% Gibco fetal bovine serum (FBS) at 5% CO_2_ and 37°C condition. The compound Olmesartan (144689-24-7) was purchased from Sigma-Aldrich, USA. The recombinant human IL-29 (1598-IL-025/CF) was from R&D Systems, USA. For the cell treatment experiment, T/C-28a2 cells were plated in 60-mm or 36-mm dishes at the density of 400,000 cells/ml media. The cells were allowed to settle overnight and reach approximately 70–80% confluency. The cells were then treated with IL-29100 ng/mL [17] with or without Olmesartan at concentrations of 1.0 and 3.0 μM [18] for 48 hours.

### Real-time PCR assay

The Trizol solution (Life, New York, USA) was used to extract total RNAs from the treated human T/C-28a2 cells, which were further transcribed into cDNA using Leukemia Virus Reverse transcriptase (Fermentas, Vancouver, Canada). The reaction was performed using the ABI 7500 real-time thermocycler (Applied Biosystems, California, USA) with the amplification condition. Real-time PCR was conducted with a LightCycler1.5 (Applied Biosystems, California, USA) and the AceQ qPCR SYBR Green Master Mix (Vazyme, Nanjing, China). Lastly, the expression of genes was determined using the 2^−ΔΔCt^ method. The following primers were used in this study: MMP-1: F: 5ʹ-ATGAAGCAGCCCAGATGTGGAG-3ʹ, R: 5ʹ-TGGTCCACATCTGCTCTTGGCA-3ʹ;

MMP-13: F: 5ʹ-CCTTGATGCCATTACCAGTCTCC-3ʹ, R: 5ʹ-AAACAGCTCCGCATCAACCTGC-3ʹ;

ADAMTS-4: F: 5ʹ- TCACTGACTTCCTGGACAATGGC-3ʹ, R: 5ʹ- GGTCAGCATCATAGTCCTTGCC-3ʹ; ADAMTS-5: F: 5ʹ-CCTGGTCCAAATGCACTTCAGC-3ʹ, R: 5ʹ- TCGTAGGTCTGTCCTGGGAGTT-3ʹ; TRAF-6: F: 5ʹ-CAATGCCAGCGTCCCTTCCAAA-3ʹ, R:5ʹ- CCAAAGGACAGTTCTGGTCATGG-3ʹ; GAPDH: F: 5ʹ-GACGGCCGCATCTTCTTGT-3ʹ, R:5ʹ-CAGTGCCAGCCTCGTCCCGTAGA-3ʹ.

### Western blot assay

Total proteins were isolated from treated human T/C-28a2 cells using the lysis buffer and were quantified using the bicinchoninic acid (BCA) kit (Vazyme, Nanjing, China), followed by being loaded onto the sodium dodecyl sulfate-polyacrylamide gel electrophoresis (SDS-PAGE). After separation for 1 h, proteins were transferred to the polyvinylidene fluoride (PVDF) membrane (Bio-Rad, California, USA) and the membrane was incubated with the primary antibody against type 2 collagen (1:500, #ab34712, Abcam, USA), Aggrecan (1:500; #216965, Abcam, USA), TRAF-6 (1:2000; #8028, Cell Signaling Technologies, USA), IκBα (1:3000; #4814, Cell Signaling Technologies, USA), p-IκBα (1:1000, #5209, Cell Signaling Technologies, USA), NF-κB p65 (1:2000; #3036, Cell Signaling Technologies, USA), lamin B1 (1:5000, #13435, Cell Signaling Technologies, USA), and β-actin (1:10,000, #3700, Cell Signaling Technologies, USA). Then, the membrane was incubated with the Horseradish Peroxidase (HRP)- linked goat anti-mouse (1:3000, #7076, Cell Signaling Technologies, USA) or goat anti-rabbit (1: 2000, #7074, Cell Signaling Technologies, USA) secondary antibodies, followed by 3 washes and exposure to ECL solution (Vazyme, Nanjing, China). Lastly, the quantification was conducted on the bands using the Image J software and normalized to the internal control β-actin or lamin B1.

### Enzyme-linked immunosorbent assay (ELISA)

The expressions of pro-form MMP-1, MMP-13, ADAMTS-4, and ADAMTS-5 were determined using ELISA assay. MMP-1 and MMP-13 kits were purchased from Elabscience, China. ADAMTS-4 and ADAMTS-5 were purchased from R&D Systems, USA. In brief, 20, 000 T/C-28a2 cells were plated on a 96-well plate. After necessary treatment, the supernatant was collected from the treated cells. The supernatant was added into the 96-well plate together with the standards to be incubated for 1 hour, followed by removing the medium and adding the conjugate solutions. After 30 minutes of incubation, the TMB solution was introduced to be incubated for 15 minutes, followed by adding the stop solution. Lastly, a microplate reader was used to measure the absorbance at 450 nm.

### 2′,7′-Dichlorofluorescin diacetate (H_2_DCF-DA) staining

The ROS level in treated human T/C-28a2 cells was determined with H_2_DCF-DA staining assay. In brief, cells were seeded on the 96-well plate, followed by being incubated with 10 μM H_2_DCF-DA at 37°C for 1 hour. Then, the fluorescence plate reader (Biotek, Vermont, USA) was used to measure the fluorescence intensity at Ex/Em = 488/525 nm.

### Superoxide dismutase (SOD) activity

The activity of SOD in treated human T/C-28a2 cells was detected using a commercial kit purchased from Sangon Biotech (Shanghai, China) in line with the described method in the previous report [19].

### Luciferase activity of NF-κB

Treated human T/C-28a2 cells were incubated for 24 hours followed by being transfected with NF-κB luciferase reporter (YEASEN, Shanghai, China) containing NF-κB response elements with the firefly luciferase gene inserted in the promoter region, with the promoterless-null Renilla construct (YEASEN, Shanghai, China) as the negative control. Lipofectamine 3000 (YEASEN, Shanghai, China) was used as the transfection reagent and the activity of luciferase and Renilla was measured using the Dual-Luciferase Reporter Assay System (Promega, Wisconsin, USA). Lastly, the luciferase activity of NF-κB was calculated after normalizing the value of luciferase activity with the activity of Renilla.

## Statistical analysis

The obtained data were expressed as mean ± standard deviation (S.D). Two-way analysis of variance (ANOVA) method with the post hoc Bonferroni correction was used to compare the difference among groups with the software of GraphPad prism 6.0. P < 0.05 was considered to be a statistically significant difference.

## Results

Using *in vitro* IL-29-challenged T/C-28a2 chondrocytes, our findings demonstrate that treatment with Olmesartan prevented the loss of type 2 collagen and aggrecan by reducing the expressions of MMP-1, MMP-13, ADAMTS-4, and ADAMTS-5. Interestingly, the protective effects of Olmesartan might be associated with its inhibitory effects on the TRAF-6/IκBα/NF-κB signaling pathway.

### Olmesartan ameliorated the degradation of type 2 collagen and aggrecan induced by IL-29 in human T/C-28a2 chondrocytes

Type 2 collagen and aggrecan are the main components of cartilage ECM, the degradation and excessive metabolism of which are regarded as the main pathological symptom of OA [20]. The expression levels of type 2 collagen and aggrecan were determined after human T/C-28a2 cells were treated with 100 ng/mL IL-29 with or without 1.0 and 3.0 μM Olmesartan for 48 hours. As shown in Figure 1, compared to the control, type 2 collagen and aggrecan were dramatically reduced in IL-29-treated human T/C-28a2 cells, which was greatly reversed by the introduction of 1.0 and 3.0 μM Olmesartan, indicating a potential protective effect of Olmesartan on disrupted cartilage ECM in OA.

**Figure 1.** Olmesartan ameliorated the degradation of type 2 collagen and Aggrecan induced by IL-29 in human T/C-28a2 chondrocytes. Cells were treated with IL-29100 ng/mL with or without Olmesartan at concentrations of 1.0 and 3.0 μM for 48 hours. (a). Molecular structure of Olmesartan; (b). Protein level of type 2 collagen and Aggrecan (***, P < 0.001 vs. vehicle group; #, ##, P < 0.05, 0.01 vs. IL-29 group, N = 5–6, two-way ANOVA).

### Olmesartan inhibited the elevated expressions of the collagenases MMP-1 and MMP-13 induced by IL-29 in human T/C-28a2 cells

MMP-1 and MMP-13 are important MMPs involved in the degradation of collagens [21]. We found that the elevated expression levels of both MMP-1 and MMP-13 in IL-29-treated human T/C-28a2 cells were significantly decreased by 1.0 and 3.0 μM Olmesartan (Figure 2a). In addition, compared to the control, the secretion of MMP-1 (Figure 2b) was pronouncedly promoted from 153.4 pg/mL to 735.8 pg/mL in human T/C-28a2 cells induced with IL-29, then greatly suppressed to 432.4 pg/mL and 253.5 pg/mL by 1.0 and 3.0 μM Olmesartan, respectively. In addition, the production of MMP-13 in the control, IL-29, 1.0, and 3.0 μM Olmesartan groups was 193.5, 857.8, 613.6, and 322.6 pg/mL, respectively. These data collectively imply that the downregulation of collagenases induced by Olmesartan might be responsible for its protective effect on ECM.

**Figure 2.** Olmesartan inhibited the elevated expression of the collagenases MMP-1, and MMP-13 induced by IL-29 in human chondrocytes. Cells were treated with 100 ng/mL IL-29 with or without Olmesartan at concentrations of 1.0 and 3.0 μM for 48 hours. (a) mRNA Level of MMP-1 and MMP-13; (b) Secretion of MMP-1 and MMP-13 (***, P < 0.001 vs. vehicle group; #, ##, P < 0.05, 0.01 vs. IL-29 group, N = 6,, two-way ANOVA).

### Olmesartan inhibited the elevated expressions of ADAMTS-4 and ADAMTS-5 induced by IL-29 in human T/C-28a2 cells

ADAMTS-4 and ADAMTS-5 are important aggrecanases involved in the degradation of aggrecans [22]. As shown in Figure 3a, the upregulated ADAMTS-4 and ADAMTS-5 in IL-29-treated human T/C-28a2 cells were significantly downregulated by 1.0 and 3.0 μM Olmesartan. The protein levels of ADAMTS-4 (Figure 3b) in the control, IL-29, 1.0, and 3.0 μM Olmesartan groups were 117.6, 504.3, 323.9, and 193.4 pg/mL, respectively. Compared to the control, the protein levels of ADAMTS-5 in IL-29-treated human T/C-28a2 cells were elevated from 134.8 to 622.5 pg/mL, then significantly decreased to 472.6 and 276.2 pg/mL by 1.0 and 3.0 μM Olmesartan, respectively. These data collectively suggest that the downregulation of aggrecanases induced by Olmesartan might be involved in the protective effect of Olmesartan on ECM.

**Figure 3.** Olmesartan inhibited the elevated expression of ADAMTS-4 and ADAMTS-5 induced by IL-29 in human chondrocytes. Cells were treated with 100 ng/mL IL-29 with or without Olmesartan at concentrations of 1.0 and 3.0 μM for 48 hours. (a) mRNA Level of ADAMTS-4 and ADAMTS-5; (b) Protein level of ADAMTS-4 and ADAMTS-5 (***, P < 0.001 vs. vehicle group; #, ##, P < 0.05, 0.01 vs. IL-29 group, N = 5–6, two-way ANOVA).

### Olmesartan alleviated the oxidative damage induced by IL-29

Oxidative damage in chondrocytes is reported to be a critical pathological change during the progression of OA [23]. We further measured the cellular ROS levels and the SOD activity in human T/C-28a2 cells following different treatment strategies. Compared to the control, the ROS level (Figure 4a) was significantly elevated and the SOD activity (Figure 4b) greatly declined in IL-29-treated human T/C-28a2 cells, both of which were dramatically reversed by incubation with 1.0 and 3.0 μM Olmesartan, indicating a potential anti-oxidative stress property of Olmesartan.

**Figure 4.** Olmesartan alleviated the oxidative damage induced by IL-29 in human chondrocytes. Cells were treated with IL-29100 ng/mL with or without Olmesartan at concentrations of 1.0 and 3.0 μM for 48 hours. (a) ROS level was detected using cell-permeable fluorogenic probes H2DCF-DA; (b) SOD level was determined (***, P < 0.001 vs. vehicle group; #, ##, P < 0.05, 0.01 vs. IL-29 group, N = 6, two-way ANOVA).

### Olmesartan inhibited the elevated expression of TRAF-6 induced by IL-29 human T/C-28a2 cells

TRAF-6 is a critical mediator for osteoclastogenesis [24] and contributes to the progression of osteoclast differentiation [25]. We found that the expression level of TRAF-6 (Figure 5a–b) was significantly elevated by IL-29 in human T/C-28a2 cells, then greatly suppressed by 1.0 and 3.0 μM Olmesartan, indicating an inhibitory effect of Olmesartan on osteoclastogenesis and osteoclast differentiation.

**Figure 5.** Olmesartan inhibited the elevated expression of TRAF-6 induced by IL-29 in human chondrocytes. Cells were treated with 100 ng/mL IL-29 with or without Olmesartan at concentrations of 1.0 and 3.0 μM for 48 hours. (a). mRNA Level of TRAF-6; (b). Protein level of TRAF-6 (***, P < 0.001 vs. vehicle group; #, ##, P < 0.05, 0.01 vs. IL-29 group, N = 6, two-way ANOVA).

### Olmesartan inhibited the elevated expression of phosphorylated IκBα induced by IL-29

The NF-κB pathway is a classic inflammatory pathway that contributes to the production of inflammatory factors, and IκBα is the natural inhibitor of NF-κB [26]. As shown in Figure 6, compared to the control, IκBα was found to be downregulated and p-IκBα upregulated in IL-29-treated human T/C-28a2 cells, both of which were dramatically reversed by 1.0 and 3.0 μM Olmesartan, indicating an inactivation function of Olmesartan on the NF-κB pathway.

**Figure 6.** Olmesartan inhibited the elevated expression of p-IκBα induced by IL-29. Cells were treated with 100 ng/mL IL-29 with or without Olmesartan at concentrations of 1.0 and 3.0 μM for 48 hours. The expression of p-IκBα and total IκBα was determined (***, P < 0.001 vs. vehicle group; #, ##, P < 0.05, 0.01 vs. IL-29 group, N = 6, two-way ANOVA).

### Olmesartan inhibited the elevated expression of nuclear NF-κB p65 induced by IL-29

We further investigated the direct effect of Olmesartan on the NF-κB pathway. As shown in Figure 7a, compared to the control, the nuclear level of NF-κB was significantly increased in IL-29-treated human T/C-28a2 cells, which was greatly reversed by 1.0 and 3.0 μM Olmesartan. In addition, the enhanced luciferase activity (Figure 7b) in IL-29-treated human T/C-28a2 cells was significantly suppressed by 1.0 and 3.0 μM Olmesartan.

**Figure 7.** Olmesartan inhibited the elevated activation of NF-κB induced by IL-29. Cells were treated with 100 ng/mL IL-29 with or without Olmesartan at concentrations of 1.0 and 3.0 μM for 48 hours. (a) The level of nuclear NF-κB p65; (b) The luciferase activity of NF-κB p65 (***, P < 0.001 vs. vehicle group; #, ##, P < 0.05, 0.01 vs. IL-29 group, N = 6, two-way ANOVA).

## Discussion

MMPs degrade the type 2 collagens and aggrecans in the ECM by resolving the peptide linkages within the target proteins. A wide range of substrates of MMPs have been found and almost all MMPs exert a degradation function on the ECM components, including aggrecans, vitreous protein, fibronectin, laminin, and collagens [27,28]. The majority of MMPs are secreted to the extracellular matrix as inactive proenzymes and, they exert their biofunction after activation, which is an amplification of the cascade sequence activation system [29]. Currently, it is reported that MMP-13, MMP-1, MMP-2, and MMP-9 are closely associated with the pathogenesis of OA [30]. We found that the degradation of type 2 collagens in IL-29-treated human T/C-28a2 cells was accompanied by the upregulation of MMP-1 and MMP-13. After treatment with Olmesartan, the degradation of type 2 collagens and upregulation of MMPs were significantly alleviated, indicating that Olmesartan prevented the degradation of ECM components by inhibiting the activity of MMPs. Type 2 collagens are the main collagens in human articular cartilage that maintain the expansion pressure of aggrecans by providing a stable structure. The ADAMTS family contributes to the disruption of articular cartilage by degrading the aggrecans [31]. In human cartilage tissues, ADAMTS-4 and ADAMTS-5 are the main ADAMTSs [32]. It is reported that the expression levels of ADAMTS-4 and ADAMTS-5 could be elevated by the inflammatory reactions induced by TNF-α [33]. In human ATDC5 chondrocytes, following stimulation with IL-1β for 3 days, cartilage degeneration is observed, accompanied by the upregulation of MMP-13 and ADAMTS-5 [34]. We found that aggrecans were significantly degraded in IL-29-treated human T/C-28a2 cells, accompanied by the upregulation of ADAMTS-4 and ADAMTS-5. Following the introduction of Olmesartan, the degradation of aggrecans and upregulation of ADAMTSs were significantly ameliorated, indicating that Olmesartan prevented the degradation of ECM components by inhibiting the activity of ADAMTSs.

Oxidative stress is an important inducer for the apoptosis of chondrocytes in the progression of OA, and is mainly induced by the excessive release of ROS that cannot be eliminated by the anti-oxidative system [23]. In the present study, we found that the activated oxidative stress in IL-29-treated human T/C-28a2 cells was dramatically suppressed by Olmesartan, indicating a promising anti-oxidative stress property of Olmesartan. In our future work, deeper investigations on the regulatory effect of Olmesartan on oxidative stress will be explored, including mitochondrial function and the Nrf2 pathway.

The NF-κB pathway is involved in the regulation of multiple cellular processes, such as inflammation, immune reactions, and stress [35]. In the classic pathway, following internal or external stimuli, the activation of IKKs is triggered to induce the degradation of IκB, further contributing to the separation of IκB from NF-κB. Separated NF-κB p65 proteins are then transferred into the nucleus to initiate the transcription of multiple cytokines, such as IL-6, IL-1β, and TNF-α. The apoptosis of chondrocytes is induced by these pro-inflammatory factors, ultimately contributing to the development of OA [7]. We found that the activation of IκB was induced by IL-29, accompanied by the increased nuclear NF-κB p65 level and enhanced transcriptional function of NF-κB, indicating that the NF-κB pathway in chondrocytes was activated by IL-29. The activated NF-κB pathway was observed to be significantly inhibited by the treatment with Olmesartan. Our future work will serve to confirm the regulatory effect of Olmesartan on the NF-κB pathway by introducing an NF-κB pathway agonist.

The limitations of the current study have to be mentioned. Although the immortalized mouse chondrocyte cell line C-28a2 has been widely used in cartilage research, it lacks some of the critical phenotypes of primary chondrocytes, and tends to lose the chondrocyte identity [36]. Therefore, the test in immortalized chondrocytes should be validated in chondrocytes in situ. Ideally, the tests in primary isolated chondrocytes from an OA patient could be used to verify the effect of Olmesartan. Secondly, the pathogenesis of OA is a complex process comprising multiple cell types and the interactions amongst them. Although chondrocytes play a critical role in OA, the involvement of other cell types and many factors should be addressed too. Therefore, the therapeutic effect of Olmesartan in OA animal models is warranted in the future. Thirdly, the regulatory mechanism of Olmesartan on NF-κB remains to be unclear, we showed that Olmesartan suppressed IL-29- induced cytosol TRAF6 induction and IκB activation. Currently, it is not clear if Olmesartan directly regulates TRAF6 or acts via the other receptor on the cell membrane. NF-κB activation plays an important role in Angiotensin II-mediated inflammation via AT2 receptors [37]. However, Olmesartan is a specific AT1 inhibitor with no antagonistic effect on AT2 [12]. Thus, the action of Olmesartan on NF-κB suppression may be independent of its effect on the AT1 receptor.

## Conclusion

In summary, our data reveal that Olmesartan exerted protective functions on IL-29- induced type 2 collagen degradation by regulating MMPs and ADAMTSs in human chondrocytes. Mechanistically, Olmesartan ameliorated IL-29-induced TRAF6/IκBα/ NF-κB activation. Our data indicate that Olmesartan may have therapeutic potential for the treatment of OA.

## Data Availability

Data of this study is/are available upon reasonable request to the corresponding authors.
